# Development and Verification of a Combined Diagnostic Model for Sarcopenia with Random Forest and Artificial Neural Network

**DOI:** 10.1155/2022/2957731

**Published:** 2022-08-23

**Authors:** Shangjin Lin, Cong Chen, Xiaoxi Cai, Fengjian Yang, Yongqian Fan

**Affiliations:** ^1^Department of Orthopeadic, Huadong Hospital Affiliated to Fudan University, Shanghai 200040, China; ^2^Shanghai Key Laboratory of Clinical Geriatric Medicine, Shanghai 200040, China

## Abstract

**Background:**

Sarcopenia is a chronic disease characterized by an age-related decline in skeletal muscle mass and function, and diagnosis is challenging owing to the lack of a clear “gold standard” assessment method.

**Objective:**

This study is aimed at combining random forest (RF) and artificial neural network (ANN) methods to screen key potential biomarkers and establish an early sarcopenia diagnostic model.

**Methods:**

Three gene expression datasets were downloaded and merged by searching the Gene Expression Omnibus (GEO) database. Differentially expressed genes (DEGs) in the merged dataset were identified by R software and subjected to Gene Ontology (GO) and Kyoto Encyclopedia of Genes and Genomes (KEGG) enrichment analyses. Afterward, the STRING database was employed for interaction analysis of the differentially encoded proteins. Then, RF was used to identify key genes from the DEGs, and a sarcopenia diagnostic model was constructed by ANN. Finally, the diagnostic model was assessed using a validation dataset, while its diagnostic performance was evaluated by the area under curve (AUC) value.

**Results:**

107 sarcopenia-related DEGs were identified, and they were mainly enriched in the FoxO and AMPK signaling pathways involved in the molecular pathogenesis of sarcopenia. Thereafter, seven key genes (MT1X, FAM171A1, ZNF415, ARHGAP36, CISD1, ETNPPL, and WISP2) were identified by the RF classifier. The proteins encoded by three of these genes (CISD1, ETNPPL, and WISP2) may be potential biomarkers for sarcopenia. Finally, a diagnostic model for sarcopenia was successfully designed by ANN, achieving an AUC of 0.999 and 0.85 in the training and testing datasets, respectively.

**Conclusion:**

We identified several potential genetic biomarkers and successfully developed an early predictive model with high diagnostic performance for sarcopenia. Moreover, our results provide a valuable reference for the early diagnosis and screening of sarcopenia in the future.

## 1. Introduction

With the aging of the population, age-related sarcopenia has emerged as a potential public health issue. Sarcopenia is generally defined as a progressive and systemic skeletal muscle disease characterized by accelerated loss of skeletal muscle mass and function, also known as muscle attenuation syndrome [1]. The loss of skeletal muscle function is an inevitable event in the normal aging process and significantly impacts the quality of life, considering it increases the risk of adverse consequences such as falls, fractures, physical disabilities, and death [2]. According to the definition of the European Working Group on Sarcopenia in Older People (EWGSOP), the prevalence of sarcopenia in European men aged 40-79 years is 1.6% and 3.66% in the elderly population (average age 85 years) [3, 4]. The World Health Organization has recognized sarcopenia as a disease since 2016, and sarcopenia was coded as M62.84 according to the International Statistical Classification of Diseases and Related Health Problems 10th Revision [5].

Recent studies have established that sarcopenia is caused by multiple complex pathophysiological mechanisms and is not solely due to nutritional deficiencies or an inactive lifestyle [6]. However, its pathogenesis has not been thoroughly explored. Most scholars postulate that aging remains the leading cause of sarcopenia. The predominant pathological features of sarcopenia are muscle fiber atrophy and increased interstitial fibrous tissue. Indeed, the decreased skeletal muscle mass in the elderly is likely due to a reduction in the size and number of muscle fibers [7]. In addition, apparent interstitial fibrosis can be observed in the skeletal muscle fibers of the elderly, which contributes to impairing the contractility of muscle fibers [8]. Aging is also associated with physiological alterations, such as motor neuron loss, mitochondrial dysfunction, age-related hormonal fluctuations, and increases in proinflammatory cytokines [9]. Nonetheless, the molecular mechanisms of these factors in the development and progression of sarcopenia remain unclear. In this study, machine learning was utilized to identify the key genes related to sarcopenia, facilitating efforts to further elucidate the molecular mechanism underlying sarcopenia caused by aging.

According to the consensus of EWGSOP, the progression of sarcopenia can be generally divided into three stages: presarcopenia, sarcopenia, and severe sarcopenia [10]. However, the current lack of a functional “gold standard” for sarcopenia diagnosis makes the screening and prevention of the disease problematic. The EWGSOP recommends using the presence of both low skeletal muscle mass and decreased skeletal muscle function as diagnostic criteria for sarcopenia. At present, there are numerous methods to assess skeletal muscle mass, including dual-energy X-ray absorptiometry (DEXA), bioelectrical impedance analysis (BIA), magnetic resonance imaging (MRI), and computed tomography (CT). Nevertheless, there is no consensus on the optimal method for measuring skeletal muscle mass, especially in clinical practice. Various physical fitness tests can be used to assess skeletal muscle function, including gait speed, 6-minute walk test, and timed stair tests. Regrettably, each method possesses its strength and weaknesses and only focus on one aspect of skeletal muscle function. Meanwhile, the Foundation for the National Institutes of Health (FNIH) Sarcopenia Project proposed a new criterion based on muscle mass, muscle strength, and physical performance to define sarcopenia [11]. Owing to the lack of diagnostic criteria for sarcopenia, it is challenging to implement screening in the elderly population. Therefore, it is imperative to discover the critical genes of sarcopenia, which will be conducive to understanding the molecular pathological process of age-induced deterioration of skeletal muscle mass and function.

In recent years, the development and application of microarray technology have made new progress in revealing the causative factors and the pathogenesis of sarcopenia. Nevertheless, the key challenge in developing diagnostic prediction models has been identifying the vital characteristic genes of sarcopenia through microarray gene expression data. Hence, various machine learning techniques, such as random forest (RF), artificial neural networks (ANN), and multivariate regression, were applied to address this problem [12, 13]. Besides, machine learning techniques are widely used, not only in medical applications but also in the field of gesture recognition [14]. Kaluri and Reddy [15] proposed a recognition algorithm with feature selection based on self-improved genetic algorithm (SIGA) to facilitate proficient gesture recognition using the machine learning techniques. With the high accuracy of the algorithms, the combination of these classification methods has made outstanding contributions to disease diagnosis and prognosis. Herein, a diagnostic prediction model of sarcopenia was developed using microarray gene expression data from the Gene Expression Omnibus (GEO) database with the combination of RF and ANN due to the extreme computational power. Firstly, the RF machine learning classifier was trained on the subset of differentially expressed genes (DEGs) from three GEO datasets to identify key genes of sarcopenia. Secondly, the weights of the key genes were calculated separately using ANN. These key genes were fed into a series of hidden layers of artificial neurons, transforming their inputs into the output layer. Finally, RF and ANN were combined to construct a diagnostic prediction model for sarcopenia. Besides, another GEO dataset was used to verify the accuracy of our diagnostic model (see the research design process in Figure 1).

## 2. Materials and Methods

### 2.1. Data Acquisition and Preprocessing

In this study, four microarray expression datasets from the National Center for Biotechnology Information Gene Expression Omnibus database (NCBI-GEO; https://www.ncbi.nlm.nih.gov/geo/) were acquired with the keywords “sarcopenia, human.” In order to obtain a larger sample size, three GEO datasets (GSE8479, GSE9103, and GSE38718) were merged as the training dataset, and GSE1428 served as the validation dataset. R software (version 4.1.3) was used to perform log2 transformation on the gene expression data of all datasets, and a Perl script (version 5.32.1.1) was used to merge the three GEO datasets into a training dataset to screen common gene probes. Besides, batch correction was conducted using the “limma” package of R software [16].

### 2.2. DEG Analysis

As presented in Table 1, the training dataset comprised 50 normal samples and 43 senile sarcopenia samples. In addition, all muscle biopsy specimens were taken from the vastus lateralis muscle. The “limma” package of the R software was used to analyze the DEGs in the training dataset. In this study, genes were considered DEGs if they met the double-filtering criterion: absolute log2-fold change > 0.5 and Benjamini-Hochberg false discovery rate (FDR)–adjusted *P* value ≤ 0.05. DEGs were visualized using the “ggplot2” and “pheatmap” packages of R software [17, 18] to generate volcano plots and heat maps, respectively.

### 2.3. Functional Enrichment Analysis and Protein–Protein Interaction

To further reveal the characteristic biological properties of DEGs, the “clusterProfiler” package in R software [19] and Metascape (http://metascape.org) were employed to perform functional enrichment analysis, including cellular component (CC), molecular function (MF), biological process (BP), and Kyoto Encyclopedia of Genes and Genomes (KEGG) pathway analysis. Terms with corrected threshold *P* < 0.05 were considered significantly enriched by DEGs. Metascape was used to visualize the output of diagrams depicting the functional interaction network between pathways. Bubble and bar charts were generated using the “ggplot2” and “clusterProfiler” packages in R to visualize Gene Ontology (GO) enrichment analysis of DEGs. Multiseries chord graphs for the top 8 KEGG terms of DEGs were created using the “ggplot2” and “GOplot” packages in R [20]. Lastly, the STRING database (https://string-db.org/) was used to analyze the protein–protein interaction network (PPI) of the DEG-encoded proteins.

### 2.4. Random Forest Screening for Key Genes

The R package “randomforest” [13] was used to screen the training dataset's DEGs for key genes. To begin, the RF model calculated the average error rate of DEGs in the training dataset to identify the optimal number of variables. Next, each error rate of 1 ~ 500 trees was calculated, and the optimal number of trees was identified based on the lowest error rate and the best stability. After determining the above parameters, a random forest tree model was constructed. Finally, the random forest classifier was used to calculate the feature importance scores, and the genes with an importance value greater than 1.5 were selected as the key genes of sarcopenia according to the Gini coefficient method. Unsupervised hierarchical clustering of key genes of sarcopenia in the training dataset was reclassified, and a heat map was created using the “pheatmap” package of R.

### 2.5. Receiver Operating Characteristic (ROC) Curve of Key DEGs

Area under curve (AUC) calculation and ROC curves were plotted for key DEGs of sarcopenia using the “pROC” package of R [21]. The diagnostic accuracy of key DEGs was evaluated by an AUC value greater than 0.7. The best cut-off of this ratio was selected according to the Youden index, and corresponding 95% confidence intervals (CIs) were reckoned with confidence interval estimation.

### 2.6. Construction of the Diagnostic and Predictive Models by ANN

First, the Min-Max normalization method was used to standardize and filter the data. Then, an ANN model of the key DEGs was built using the “neuralnet” package of R [22], and the processed training data was fed into the ANN model. Five hidden layers and two outputs (normal and sarcopenia) were set as model parameters. Finally, the sum of the disease classification score was calculated by multiplying the weight score by the expression level of each gene. The ROC curve of the training set was drawn using the “pROC” package of R to calculate the area under the curve (AUC) for assessing the accuracy of the ANN model.

### 2.7. ANN Model Verification

To evaluate the diagnostic performance of the ANN model, an external dataset (GSE1428) was used as a test dataset to validate the diagnostic and predictive model. The ROC curve of GSE1428 was generated using the “pROC” package of R, and the AUC and 95% CI were used to validate the efficiency of the model.

## 3. Results

### 3.1. Screening of DEGs

107 DEGs were identified between 43 senile sarcopenia and 50 normal samples in the training dataset using the “limma” package of the R software. DEGs included 46 lowly expressed genes and 61 highly expressed genes, including SLPI and MYH8 with log FC > 1. The results of DEGs were visualized in the volcano map and heat map (Figure 2). Details of the DEGs are provided in Supplementary file 1.

### 3.2. GO and KEGG Enrichment Analyses of the DEGs

GO enrichment analysis of the DEGs yielded 242 enriched annotations, including 199 BPs, 31 CCs, and 12 MFs. The top five most significant GO terms of BP, CC, and MF are illustrated in the bubble and bar charts (Figures 3(a) and 3(b)). DEGs were primarily enriched in the development of muscle tissue and organs, the stress response and detoxification of copper ions, and animal organ regeneration in the BP category. They were mainly enriched in the complex of muscle myosin and myosin II, myofibril, contractile fiber, and myosin filament in the CC category. Among the MF category, DEGs were mainly enriched in the structural constituent of muscle and binding of peptide, tau protein, muscle alpha-actinin, and unfolded protein. Moreover, KEGG pathway enrichment analysis was also performed on the DEGs. The results showed that the DEGs were mainly enriched in the transcriptional misregulation in cancer, FoxO signaling pathway, AMPK signaling pathway, glucagon signaling pathway, and regulation of glucose metabolism (see Table 2 for details). Figures 3(c) and 3(d) delineates the top five most significant KEGG terms and the crucial DEGs involved in the pathways. Based on the module analysis of the PPI network, a total of 101 protein–protein interaction pairs involving 71 proteins were acquired (Figure 4(a)). Details of the analysis results of PPI networks are listed in Supplementary file 2. In addition, Figure 4(b) also depicts the interaction network between GO terms and KEGG pathways.

### 3.3. Screening for Key DEGs by Random Forest

107 DEGs were input into the RF classifier, and the optimal mtry parameter was set (specifying the optimal number of variables considered at each split of regression trees). Then, recurrent random forest classification was carried out on all possible numbers in the 1-107 variables, and the average error rate of the model was subsequently calculated. Next, we selected 115 trees as the parameters of the final model, according to the relationship between the model error and the number of decision trees (Figure 5(a)) to demonstrate the stable error in the RF model. The importance of variables (Gini coefficient method) was measured to lower the accuracy and mean square error of the output during the construction of the RF model. Finally, seven DEGs with an importance value greater than 1.5 were identified as key genes in sarcopenia (Figure 5(b)).

### 3.4. Heap Plot and ROC Curve of Key DEGs

*K*-means clustering was performed on the training dataset without supervision based on these seven critical variables. The heat plot (Figure 6(a)) showed that the 93 samples of the training dataset converged perfectly in the healthy and sarcopenic groups, which meant that the seven key genes could be used to distinguish sarcopenia from healthy samples. ROC curves of the seven key genes were plotted, and the AUC was calculated for each gene (Figure 6(b)). The order of efficacy evaluation of these seven genes in diagnosing sarcopenia was MT1X, FAM171A1, ZNF415, ARHGAP36, CISD1, ETNPPL, and WISP2, as listed in Table 3.

### 3.5. Construction and Verification of the ANN Model

Vital genes that best differentiate sarcopenia from normal samples were identified using RF classifiers during the construction of the RF model. The first step of constructing the ANN model was data preprocessing for normalized data. Then, a specific scoring model for sarcopenia was established by calculating the weights for each gene through artificial neural network analysis. The ANN topology of the training dataset included seven input layers, five hidden layers, and two output layers. The neural network weight scores for each gene are detailed in Supplementary file 3. Based on the above, we constructed an ANN model of sarcopenia for classifying gene expression data between sarcopenia and normal samples via the “neuralnet” package of R (Figure 7). The area under the ROC curve was used to evaluate the classification performance of the model. The model predicted an AUC of 0.999 in the training dataset (Figure 8(a)) and 0.85 in the test dataset (GSE1428) (Figure 8(b)), indicating that the ANN model had high classification performance. The aforementioned results demonstrated that a diagnostic model for sarcopenia was successfully constructed from the differential gene expression of sarcopenia and normal samples.

## 4. Discussion

Declining muscle mass and function in older adults is a major health concern; thus, early prediction and diagnosis of sarcopenia can increase the odds of intervention. However, the definition of sarcopenia has only been established in recent years. More importantly, there is no internationally accepted standard for the diagnosis of sarcopenia. Therefore, establishing an early diagnostic screening model that may aid in identifying characteristic biomarkers of sarcopenia is essential. We did not focus on phenotypic diagnosis but instead constructed a gene-level diagnostic model of sarcopenia using machine learning methods that have shown significant advantages in gene selection and classification. In recent years, improvements in machine learning techniques and the availability of gene expression data in public databases have provided new diagnostic and predictive options for sarcopenia.

In this study, we collected microarray expression profiling datasets from the GEO database (GSE8479, GSE9103, and GSE38718) and obtained 107 DEGs between sarcopenic and normal muscle samples. RF screening was performed on 107 DEGs, and 7 signature genes were identified between sarcopenia and normal groups. The ANN model was used to calculate the predictive weight of the seven signature genes. Thereafter, a classification scoring model for sarcopenia was also developed, and the classification effect of the model was evaluated. In addition, we compared the established diagnostic model in terms of predictive accuracy in the training and testing datasets using the AUC of ROC curves, and the results revealed that our established model had high diagnostic power. To our knowledge, this is the first study to construct a diagnostic model for sarcopenia.

To begin, the research identified 107 DEGs through bioinformatics analysis of 93 muscle samples in the GEO database. Notably, the expression levels of SLPI and MYH8 in the sarcopenia group were significantly higher than those in the normal group (log2 FC > 1). A secretory leukocyte peptidase inhibitor (SLPI) is encoded by the SLPI gene, serving as an inhibitor of nuclear factor-*κ*B (NF-*κ*B), which can bind to IL-8 and tumor necrosis factor-*α* (TNF-*α*) sites on the promoter [23]. NF-*κ*B, as a family of nuclear inflammatory transcription factors, is activated by TNF-*α* in skeletal muscle cells to regulate muscle metabolism [24]. High expression of myosin heavy chain 8 (MYH8) is a marker of muscle regeneration [25]. As a component of myosin, MYH8 is chiefly expressed in neonatal skeletal muscles [26]. In certain pathological states, progenitor cells can proliferate and differentiate into muscle cells during skeletal muscle regeneration but fail to develop during the fiber maturation stage [27]. Regrettably, the random forest classifier did not identify SLPI and MYH8 as candidates for the diagnostic model.

The pathogenesis of sarcopenia is complex, and its molecular mechanism involves the regulation of multiple cellular signaling pathways. Generally speaking, key genes, signaling pathways, and PPI networks govern muscle hypertrophy and atrophy information individually or in combination, maintaining a balance between protein synthesis and hydrolysis. The GO enrichment results were presented as bar and bubble graphs in this study. As illustrated in Figure 3, among the top 15 most important GO terms, nine terms were related to skeletal muscle maintenance and development, including muscle structural components, myosin and myosin II complexes, contractile fibers, and myosin filaments. Interestingly, we also found two GO terms implicated in the stress response and detoxification of copper ions. These results led us to speculate that copper ions might accumulate in skeletal muscle cells of sarcopenic patients. Recent studies have reported that copper ions are directly bound to fatty acylated components in the tricarboxylic acid cycle pathway, resulting in an aberrant aggregation of fatty acylated proteins and loss of iron-sulfur cluster proteins, eventually leading to cell death [28]. Therefore, cell death induced by copper ions may be a pivotal mechanism behind the occurrence and development of sarcopenia, which warrants further studies. According to the KEGG pathway enrichment analysis (Table 2), AMPK and FoxO signaling pathways were the two pathways closely related to the pathogenesis of sarcopenia. AMP-activated protein kinase (AMPK), associated with the regulation of multiple cellular functions, is a crucial regulator of skeletal muscle mitochondrial function and oxidative stress [29]. Activated AMPK can modulate energy metabolism-related pathways, promote mitochondrial biogenesis, and improve skeletal muscle dysfunction during aging [30]. As the intracellular energy factory generating ATP for muscle contraction, the mitochondria play a fundamental role in the pathogenesis of primary sarcopenia. Therefore, regulating mitochondrial respiratory function may be one of the ways by which the AMPK signaling pathway maintains skeletal muscle mass. The FoxO signaling pathway is one of the most critical cellular signaling pathways in skeletal muscle proteolysis. Forkhead box transcription factors (FoxO) are widely distributed in various eukaryotes, including FoxO1, FoxO3a, and FoxO4 in skeletal muscle [31]. FoxO1 and FoxO3a proteins transcriptionally upregulate the expression of the muscle-enriched E3 ubiquitin ligase closely related to muscle atrophy, including muscle RING finger 1 (MuRF1) and muscle atrophy F-box (MAFbx) [32]. The FoxO transcriptional network not only accelerates the activation of the ubiquitin-proteasome system (UPS) but also activates the autophagy-lysosome system responsible for degrading misfolded proteins and organelles, especially mitochondria [33]. UPS, together with autophagy, induces skeletal muscle protein breakdown by increasing protein degradation and expanding the binding of ubiquitin to muscle proteins, signaling that this cellular signaling pathway plays an essential role in the pathogenesis of sarcopenia.

In this study, DEGs related to sarcopenia were identified through gene expression differential analysis. Afterward, seven key DEGs were identified through the random forest classifier, and a distinct diagnostic model for sarcopenia was established for the first time through neural network models. MT1X showed the highest diagnostic performance among these seven genes according to the AUC of the ROC curve. MT1X encodes metallothionein-1X, a functional (sub) isoform of MT1 encoded by genes located on chromosome 16q13 [34]. Metallothionein is a small metal-binding protein rich in cysteine and plays a nonnegligible role in maintaining metal homeostasis in cells and transition metal detoxification [35]. MX1X overexpression in skeletal muscle of the elderly suggests the presence of overloaded deposition of metal ions, such as iron and copper ions, involved in the development and progression of sarcopenia. Besides, previous studies have described that dexamethasone can induce an upregulation in the expression of MX1X in human tracheal smooth muscle cells [36]. Interestingly, dexamethasone also causes skeletal muscle atrophy due to the loss of fast fibers (type II), similar to muscle fiber variations in primary sarcopenia caused by aging [37].

Surprisingly, during the analysis to construct the diagnostic model of sarcopenia, three key genes (CISD1, ETNPPL, and WISP2) that might play a vital role in the pathogenesis were identified for the first time. CDGSH iron-sulfur domain 1, encoded by CISD1, is an iron-containing mitochondrial outer membrane protein regulating mitochondrial iron uptake and respiratory capacity [38]. CISD1 deficiency induces excessive iron accumulation in the mitochondria, resulting in mitochondrial dysfunction and subsequent oxidative stress damage [39]. Furthermore, the heat map of key DEGs (Figure 6(a)) revealed that the expression of CISD1 in the sarcopenia group was significantly lower than that in the normal group, indicating that iron overload might be present in the mitochondria of skeletal muscle cells of sarcopenic patients. Therefore, we speculated that the imbalance of iron homeostasis caused by the decreased expression of CISD1 might be implicated in the pathogenesis of sarcopenia. Ethanolamine phosphate phospholyase (ETNPPL), previously referred to as Agxt2l1, is a gene encoding the Etnppl protein, which was discovered to specifically and irreversibly degrade phosphoethanolamine (PETN) [40]. In addition, PETN was found to be a potent inhibitor of mitochondrial respiration [41]. Therefore, we postulated that ETNPPL maintained mitochondrial respiration and energy production. In this study, the expression of ETNPPL was significantly lower in sarcopenia samples than in normal samples, which indirectly supported our hypothesis. WNT1-inducible-signaling pathway protein 2 (WISP2) encoded by WISP2 is a novel adipokine, most highly expressed in the adipose tissue [42]. Studies on the secretome of human adipose tissue have determined that WISP2 is the protein most differentially secreted between obese and lean individuals [43]. As is well documented, the leading cause of insulin resistance and type 2 diabetes is obesity. Significant changes in body composition with age include increased body fat and decreased skeletal muscle. Therefore, sarcopenic obesity was first defined in 2000 as the co-presence of sarcopenia and obesity [44]. Herein, the expression of WISP2 in sarcopenia samples was significantly higher than that in normal samples, suggesting that this highly expressed secreted adipokine might be a risk factor for sarcopenic obesity.

Despite the innovative findings, there are still several limitations that need to be considered. Firstly, the training dataset combined three small sample size datasets. Although the batch effect was removed, it was still not the most appropriate dataset. Therefore, this diagnostic model needs to be continuously validated and revalidated using independent datasets with a larger sample size in the future. Secondly, the difficulty in obtaining muscle specimens may limit the clinical application of this diagnostic model. Thirdly, our sarcopenic prediction model was constructed based on datasets from the GEO database, and future studies will require in vitro and in vivo experiments to practice and validate the predictive model. However, the proteins encoded by these key genes identified in this study have the potential to become characteristic biomarkers of sarcopenia, laying the foundation for the diagnosis and screening of sarcopenia in the future.

## 5. Conclusion

In this study, seven genetic biomarkers closely associated with sarcopenia, such as CISD1, ETNPPL, and WISP2, were identified by RF and were used to construct a diagnostic prediction model for sarcopenia with high diagnostic performance. Furthermore, this study provides a valuable reference for the early diagnosis of sarcopenia, new hypotheses for the pathogenesis of sarcopenia, and promising predictive biomarkers for the screening of sarcopenia. Nevertheless, further studies on the molecular mechanisms in which seven genetic biomarkers are involved are still needed to validate the roles of these genes in sarcopenia.

## Figures and Tables

**Figure 1:** Flow chart of the research design.

**Figure 2:** (a) Volcano plot of DEGs. The red dots in the upper right part represent upregulated DEGs. The green dots in the upper left part represent downregulated DEGs. The middle black dots represent the remaining stable genes. (b) Heat map of DEGs. The colors from red to blue in the figure represent the expression of DEGs from high to low.

**Figure 3:** Functional and pathway enrichment analyses of DEGs in sarcopenia. (a) Bar graph of GO terms enriched in the biological process (BP), cellular components (CC), and molecular function (MF). The *X* axis represents the *q* value (−Log10), and the *Y* axis represents the GO term. (b) Bubble graph of GO term enrichment results. The *X* axis represents the gene ratio, and the *Y* axis represents the GO term. The size of the bubble represents the number of DEGs enriched in the GO terms. (c) Chord plot showing KEGG pathways. DEGs are indicated on the left. The different colored bands on the right represent different KEGG pathways. Connecting lines indicate that the gene is enriched in the KEGG pathway. (d) Circle plot showing KEGG pathways. The circle inside represents DEGs, blue represents downregulated DEGs, and red represents upregulated DEGs. The outer circle represents different KEGG pathways.

**Figure 4:** (a) Protein–protein interaction network analysis of the DEGs. (b) The interaction network between GO terms and KEGG pathways. Different colored nodes represent different GO terms or KEGG pathways.

**Figure 5:** (a) The influence of the number of decision trees on the error rate. The *X* axis indicates the number of decision trees, and the *Y* axis represents the error rate. (b) Results of the Gini coefficient method in random forest classifier. The *X* axis represents the importance index, and the *Y* axis represents the gene name.

**Figure 6:** (a) Heat map of seven key DEGs in sarcopenia. The colors from red to blue in the figure represent the expression of key DEGs from high to low. (b) ROC curves of seven key DEGs. Different colored curves represent different genes.

**Figure 7:** Results of neural network visualization.

**Figure 8:** ROC curves of the ANN diagnostic model of sarcopenia. (a) AUC validation results of the ANN model on the training dataset. (b) AUC validation results of the ANN model on the testing dataset.

**Table 1:** Source of GEO datasets.

GEO datasets	Platform	Sarcopenia samples	Normal samples
Train group			
GSE8479	GPL2700	25	26
GSE9103	GPL570	10	10
GSE38718	GPL570	8	14
Test group			
GSE1428	GPL96	12	10

**Table 2:** KEGG-pathway analysis of DEGs.

KEGG	Gene symbol involved in the pathway	Count	*P*.adjust
Mineral absorption	MT1H/MT1X/MT2A/ATP1B4	4	0.00054
Glucagon signaling pathway	FOXO1/PKM/PRKAG1/FBP2/CALML6	5	0.00059
Longevity regulating pathway-multiple species	CRYAB/FOXO1/HSPA2/PRKAG1	4	0.00065
AMPK signaling pathway	FOXO1/PRKAG1/SCD/FBP2/STRADB	5	0.00099
Thyroid hormone signaling pathway	ACTB/FOXO1/MYH6/RXRG/ATP1B4	5	0.00103
Transcriptional misregulation in cancer	BCL6/CDKN1A/CEBPB/FOXO1/RXRG/GADD45G	6	0.00137
FoxO signaling pathway	BCL6/CDKN1A/FOXO1/PRKAG1/GADD45G	5	0.00147
Thyroid cancer	CDKN1A/RXRG/GADD45G	3	0.00168
Insulin signaling pathway	FOXO1/PRKAG1/FBP2/SOCS2/CALML6	5	0.00179
Carbon metabolism	GOT1/PKM/FBP2/SUCLA2	4	0.00683

**Table 3:** Evaluation of key DEG diagnostic capabilities.

Genes symbol	Sensitivity (%)	Specificity (%)	AUC	95% CI	Youden index
MT1X	0.93	0.84	0.932	0.880-0.983	0.77
FAM171A1	0.837	0.94	0.929	0.874-0.985	0.777
ZNF415	1	0.66	0.925	0.875-0.974	0.66
ARHGAP36	0.791	0.96	0.91	0.851-0.969	0.751
CISD1	0.93	0.88	0.905	0.834-0.976	0.81
ETNPPL	0.86	0.86	0.893	0.823-0.964	0.72
WISP2	0.698	0.96	0.86	0.784-0.936	0.658

## Data Availability

The data used to support the findings of this study are available from the corresponding author upon request.

## Supplementary Materials

Supplementary Materials Supplementary file 1: details of DEGs. Supplementary file 2: details of the analysis results of PPI networks. Supplementary file 3: the neural network weight scores for each gene.
